# Application of Punitive Damages in Intellectual Property Law in Complex Network Environment

**DOI:** 10.1155/2022/4806045

**Published:** 2022-09-09

**Authors:** Xiangming Mu

**Affiliations:** ^1^Southwest University of Political Science & Law, Chongqing 401120, China; ^2^Henan University of Technology Law School, Zhengzhou 450001, China

## Abstract

Many IP (intellectual property) will also be infringed, and it will become more and more serious, causing huge economic losses to people or groups who own IP. If punitive damages can be made for intentional but intentional infringement of IP, it will help to stop intentional infringement of IP, and it can also give due compensation to the obligee's loss. Based on this, this paper analyzes the introduction and implementation of punitive damages in IP law. In this paper, a relatively efficient text classification method is realized by using the method of deep learning and model design. Similar texts in the training set are grouped into a group, and each group is considered as a common text vector. Then, a threshold is set to deal with clusters higher than the threshold, and the training set is reformed. Through the experimental results, the feature extraction effect of this model is improved, the classification accuracy is constantly improved, and the final convergence rate of this model reaches 95%. It has been verified that the system can realize the automatic classification of basic Chinese patent texts.

## 1. Introduction

Punitive damages are a useful tool for both preventing and dealing with international intellectual property (IP) infringement. In order to establish the validity and necessity of punitive penalties as a form of product liability, scholars explored the history of the punitive damage system as well as its nature and function. Due diligence should therefore be exercised when applying the punitive damage system in the field of intellectual property, not only to prevent overzealous punishment and the impediment of innovation but also to address the social phenomenon of “serious infringement” and “low compensation” in China. In the recent past, a robust system for compensating IP infringers not only indicates and demonstrates the economic and legal systems' maturity, but it also effectively fosters innovation and growth in the fields of business, science, and culture.

China has always followed the principle of compensation in civil damage compensation, emphasizing that compensation is the same as damage, and the compensation that the victim gets can only be direct loss. In accordance with the principle of “whoever claims it, whoever proves it,” the amount of loss must be proved by the victim [1]. In addition, IP has certain duplication. If IP is distributed by infringers, all people who have the right to know will become infringers passively, which is a great loss to the victims. The fragmented design of the system leads to insufficient coordination of laws and regulations, and the strict application conditions and narrow application scope of the system also greatly limit the exertion of the “punitive” function [2, 3]. Lufkin thinks that “indirect intention” and “direct intention” are basically the same in terms of cognitive factors, and both of them indicate that they do not exclude the criminal result in terms of will factors [4]. Feng and Ma proposed that punitive damages should be introduced into the IP infringement compensation system in China to curb the current rampant infringement [5]. In this regard, some scholars have pointed out that the trial has the purpose of deterrence and punishment. In France, lawyers and academics generally believe that French courts sometimes use the behavior of criminals as the standard for awarding damages, in order to punish criminals for deliberately ignoring the interests of plaintiffs. Therefore, we cannot help wondering whether the above legislation with punitive damages is really punitive damages. Since then, the topic has returned to what punitive damages are, the legitimacy and necessity of punitive damages.

IP infringement occurs in all countries, and its characteristics and ways vary from country to country. Punitive damages can play a role that compensatory damages cannot and can make more adequate remedies for the victims' injuries. For example, different countries have different considerations about the purpose of punitive damage system, the way of awarding punitive damages, and the factors considered when determining the amount of punitive damages. In view of this situation, this paper chooses the subjective and intentional determination of punitive damages in IP field. Sum up the punitive liability of judicial application in China. Restrict the discretion of judges, effectively protect the legitimate interests of patentees, and increase the predictability of the law.

The innovation of this paper:

1. This paper demonstrates the legitimacy basis of IP punitive damage system from various angles, puts forward systematic legislative suggestions on China's IP punitive damage system, and probes into the reasons why they can be regarded as “subjective malice”, to be able to see the big from the small
2. Aiming at the task of Chinese patent text classification, this paper deeply studies the related technologies of each stage of text classification and designs a Chinese patent text classification system, which can systematically complete the task of Chinese patent text classification. Show the data in various charts, and users can customize the chart form

## 2. Related Work

### 2.1. Principle of IP Punitive Damages

China's current laws in the IP field have not stipulated the punitive damage system, but in practice, some basic principles to solve the problem and the main methods to calculate the compensation amount have been established. Deductions, the value of the parts themselves, and their value in the finished product profits: these factors are difficult to make an accurate judgment only by the existing knowledge and skills of the judges of the people's courts.

Yong pointed out that the applicable general conditions of tort liability are as follows: the accused infringer is at fault subjectively, the obligee suffers actual damage, and there is patent infringement [6]. Abbott described the indirect losses suffered by the patentee as follows: first, the losses are some available future benefits, only the possibility of acquiring property, not the actual benefits; secondly, this loss of future interests has practical significance, rather than abstract or hypothetical significance [7]; Cb et al. introduced the punitive damage system for product quality infringement but established the legal term of “punitive damages” [8]. Hamill believes that “knowing” can be broadly interpreted, including intentional and gross negligence [9]. Some scholars also believe that the understanding of “knowingly committing crimes” in this paper may be based on the original intention of legislators, that is, to punish those producers and operators who are subjective and malicious [10].

Qiu and Palomar think that compared with compensatory tort compensation system, the unique punitive and deterrent functions of punitive damage system are the important reasons for introducing this system [11]. Abbas et al. put forward a quasicriminal system, arguing that punitive damages in civil cases are similar to fines in criminal cases, but they are not handed over to the state treasury, but paid to individuals [12]. Graves proposed that punitive damages should be explained from the angle of economic law, which has the attributes of public law and private law, and believed that punitive damages should be the responsibility of economic law [13]. The purpose of economic law is to compensate market failure and government failure, and to safeguard social public interests in social and economic activities.

### 2.2. Research on Classification of Patent Information

Extracting information from patent texts originated in Europe, the United States, and Japan. China's patent investigation started late, but with the rapid development of the times and the rapid progress of science and technology, the importance of patent investigation has become increasingly prominent. Moreo et al. deeply studied the content level of patent text and extracted the actual content of patent text, including title, abstract, and background summary [14]; Esuli et al. put forward an automatic patent classification method based on statistical distribution and analyzed patents. According to the characteristics of text data, two metrics were added to the patent text: the interclass dispersion weight factor and the position weight factor. Experience shows that this method can achieve better classification performance [15]. Liu and Guo, based on the semantic theory, put forward the automatic abstraction technology of patent documents, which provided the foundation for the display and sharing of patent knowledge [16]. Wang and Mao used the patent extraction algorithm based on semantic and keyword statistics and achieved good experimental results [17].

Feng et al. proposed an open source word2vec toolkit for word vector pretraining, and put forward a variety of methods to optimize the training speed [18], such as negative sampling. The appearance of word2vec is a milestone in the process of text assignment, and it has been recognized by all circles. By using LSTM (long-short-term memory) to capture the dependence on context, the feature information of the text that depends on the context information is obtained, which improves the classification accuracy to a certain extent. Cunha et al. combined the results of CNN (convective neural network) and RNN (recurrent neural network) in irony pragmatic discrimination, and the classification results were better than those of a single model [19]. Wang et al. proposed an optimized KNN (*k*-nearest neighbor) algorithm classifier. The classification module consists of training, classification, and evaluation. It is found that compared with the traditional KNN algorithm, the optimized KNN algorithm has a certain degree of improvement in classification effect [20].

## 3. Methodology

### 3.1. Legislative Design of IP Punitive Damage System

The applicable conditions of IP punitive damages refer to the preconditions that the court must have to apply punitive damages to infringers in IP infringement disputes. Only when IP infringement is intentional can punitive damages be applied to infringers, which is one of the necessary conditions for applying IP punitive damages. Arbitrary behavior is lighter than intentional damage, and the subjective state of the perpetrator is lighter. Intention is a kind of knowing that there will be some kind of danger and hoping (direct intention) or allowing (indirect intention) this danger to happen. Therefore, it is considered that at least it must be proved that objective reckless behavior can be proved to be intentional infringement, to allow the damage to be aggravated.

In copyright infringement disputes, the court may order the infringer to compensate the losses of the obligee and the interests gained by the infringer due to the infringement. After determining the above two amounts, the court can still order the infringer to pay compensation to the infringer according to the circumstances of the infringement, and the infringee shall bear punitive damages. The amount of punitive damages should be determined effectively in advance, which can not only serve as compensation and warning but also should not be too large. Similar to the presumption of “knowing” in the civil law system, most judicial interpretations in the criminal law system also regard the act of “continuing to violate the law after receiving an illegal notice” as one of the manifestations of the presumption of guilty conscience of the criminal. While making up for the deficiency of the principle of punitive damages, we should give full consideration to the coordination of social public interests and personal interests, because in a broad sense, punishing offenders is to protect more potential victims, which is also a manifestation of social public interests and personal interests.

Judging from the patent laws of most countries, the fault elements of liability for compensation include intention and negligence, that is, the infringer intentionally or negligently infringes the interests of the patentee. Objectively speaking, intention is a kind of behavior that “the actor knows that he has certain civil obligations to others, but still violates this obligation, causing damage to others.” Adhering to the subjective theory does not mean giving up the method of judging the subjective mentality of the perpetrator by objective facts. The standard of “objective reckless behavior” greatly improves the identification standard of intentional misconduct, exempting the accused from the duty of care and the positive duty of obtaining counsel's opinions to defend intentional misconduct. This significantly improves the ability of patent holders to bear punitive damages.

However, at this stage, the demonstration of the direct stipulation of recidivism in Chinese legislation still needs further exploration. First, grasp the concept of recidivism, and define the difference between the concepts of “recidivism.” The calculation method of royalty multiples is also punitive. According to the original patent law, damages can be determined according to the “multiple” of the patent license fee. Defining the punitive factors in the existing patent infringement compensation system will help us better understand the patent infringement compensation system, scientifically identify the nature of the infringement compensation and make appropriate distinctions, and help to eliminate the inherent contradictions in the patent infringement compensation system.

Statistics-based methods mainly rely on large-scale corpora to calculate the probability distribution of lexical context information, which is used to calculate the semantic similarity between words. Generally speaking, a semantic dictionary constructs all the words of a language in one or more hierarchical tree diagrams and calculates the similarity between words according to the path distance between words in the diagrams. If two basic sememes are located in the same tree structure, the semantic similarity can be expressed by the distance between them. The up-down relation structure of basic sememes constitutes the basis of semantic similarity calculation.

As sememes form a tree-like structure according to the hyponymy, it can be calculated by the distance between sememes in this structure. The semantic distance between sememes is expressed by the following formula:

(1) $$\begin{array}{c} \text{Sim}\left(p_{1},p_{2}\right)=\frac{\alpha }{d+\alpha }, \end{array}$$

where *p* represents sememes, *d* represents the path length between sememes, and *α* is an adjustable parameter.

When text exists as a vector, similarity is represented by the distance between two vectors. The similarity between vectors can be calculated using many formulas. Usually, the distance between text vectors is calculated by the inner product or cosine of the angle between them. The calculation formula is as follows:

(2) $$\begin{array}{c} \text{Sim}\left(D_{1},D_{2}\right)=\overset{n}{\underset{k=1}{\sum }}w_{1k}*w_{2k}, \end{array}$$

where *w*_1*k*_, *w*_2*k*_, 1 ≤ *k* ≤ *n* is the weight of each feature item in document *D*_1_, *D*_2_ and *n* is the total number of features.

When each data arrives, it can be classified by using the constantly updated weight vector *w*_*n*+1_ at this time. On the other hand, through theoretical processing, it is found that the vector effect calculated by the average weight will be better, namely,

(3) $$\begin{array}{c} w=\frac{1}{n}\overset{n+1}{\underset{i=1}{\sum }}w_{i}. \end{array}$$

The key problem lies in the extraction of case description information. As the case description is usually expressed in natural language in our daily life, the expression is more casual, and it can be popularized in some places, which may not conform to some grammatical rules. In the process of testing, it is found that it is very difficult to accurately extract key information from the case description, which seriously affects the accuracy of legal clause retrieval. Therefore, some improvements to the original design can be considered to achieve better results. The legal support system is shown in Figure 1.

Extract words related to the legal field from legal clauses and establish a legal dictionary. For each law, extract the key words that express illegal acts from the law. Calculate the semantic similarity between the keywords expressing illegal acts in the law and the facts of the case, and judge whether illegal acts appear in the description of the case. If it appears, issue the corresponding legal provisions, and finally, get the recovery result. A kind of crime described in a clause usually contains various words that describe the behavior and the object of the behavior. In this way, for a given clause, all the words describing the behavior and the objects of the behavior in the clause are combined together, and each group expresses the illegal behavior corresponding to the clause.

In the case of trademark infringement, if the infringer infringes a well-known trademark, it is more likely to be regarded as subjective “malice” by the court. People should “know” well-known trademarks in this field. After the court knew the business secret of the partner because of cooperation, the infringement was presumed as subjective malice. The author thinks that it conveys a kind of emotion—that is, it is a kind of malice to intentionally violate the business ethics under the knowing knowledge.

Punitive damages under intellectual property law differ from standard civil damages in the criteria for fault mode. Determining the type of the infringer's error is necessary for determining whether IP infringement is intentional or not. Therefore, we can only fully comprehend the applicable criteria of PI punitive damages by correctly defining fault and intention and correctly identifying them. In other words, it describes the actor's subjective condition as manifested in their behaviour, which contravenes morality and the law. However, objective standards are typically used to evaluate negligence.

### 3.2. Large-Scale Patent Classification

To some extent, patents reflect the level and direction of scientific research in today's society. Through patent analysis, relevant information can be extracted from relevant countries, regions and economies, and automatic classification of patent texts is of great significance and practical value. It can be continuously improved by accumulating training data for a long time. This is the only way to improve the recall rate and search accuracy. In a word, it is of great practical value to classify patents and extract useful information from them.

As a specific technical asset, patent right is intangible. Although it is relatively simple and clear to judge whether patent infringement is established, it is extremely difficult to judge and evaluate the damage degree of patent right. In the current judicial practice, it is difficult to determine the compensation for patent infringement, and the applicable proportion of legal compensation is high. If this problem cannot be solved, giving judges the discretion to apply punitive damages cannot stop the system in the patent field from being rarely applied as the practice of this system in China's trademark law and the purpose of introducing and designing the patent system.

The actual loss of the right holder must be compared with the gains that the right holder can get in the ideal state of noninfringement. Therefore, the calculation is often based on the loss of income suffered by the patentee due to infringement. For example, the patentee sells items related to the patented product, but if the infringer also sells related products or series of products, the possibility of customers buying the patentee's related products will be reduced, resulting in the patentee losing the patent right.

Chinese punctuation marks are used as separators. In Chinese texts, words are the smallest units of Chinese semantic expression. Therefore, the first step to classify Chinese texts is to preprocess them, that is, to segment them first. Chinese text segmentation is to divide the text stream into words according to certain spacing rules. The quality of the data set will have a great impact on the classification results, among which the long and inconsistent length of the text makes the feature dimension of the text very high, which will bring great computational overhead and data dimension disaster, so it is necessary to reduce the feature dimension of the text. In the classification system, a threshold can be defined. If the information gain of the feature word exceeds the threshold, the feature word is selected; otherwise, the feature word is filtered.

The main idea of KNN algorithm is the *k* similar samples with the highest correlation degree. For each sample to be classified, extract its feature vector, calculate the correlation distance between it and the known data, and define the threshold. In the algorithm described in this section, the Euclidean distance formula is used to calculate the distance between sample items, and the definition formula is as follows:

(4) $$\begin{array}{c} d\left(x,y\right)=\sqrt{\overset{n}{\underset{k=1}{\sum }}{\left(x_{k}-y_{k}\right)}^{2}}. \end{array}$$

Hyperplane segmentation is a simple grouping segmentation method. The hyperplane segmentation strategy considers the spatial distribution of samples, selects a main direction in the feature space, and then, segments the samples by using the hyperplane perpendicular to the direction, so that the samples with close distance in the feature space are divided into the same subset. The formula for calculating the sample mean and covariance matrix is as follows:

(5) $$\begin{array}{c} \mu =E\left(x\right),\\ C=E\left(x-\mu \right){\left(x-\mu \right)}^{T}. \end{array}$$

The basis of Chinese patent text classification system is the storage and management of Chinese patent text data. It focuses on learning and training the patent text classification model and adjusting the parameters of the model; visualization is the key, which is beneficial to the classification of results and the effective management of patent text data in patent examiners. The main function is to visualize patent data in various forms and different dimensions. The main user is patent examiners, and patent examiners can further integrate patents according to the displayed results.

This section designs the functions of Chinese patent text classification system, which mainly includes user management module, classifier module, patent application module, and result display module. The main function is classifier module, including data preparation, text preprocessing, text rendering, and function training model. The functional architecture diagram of the system is shown in Figure 2.

Patent text is the support for the registration of patented technology. The research on its evolution can be divided into three aspects: one is the change of theme intensity in time interval, the other is the change of theme content in time interval, and the third is the change of popularity. In the patent technology of time period, there are many subjects without obvious semantic information. On the contrary, if the number is too small, a topic will contain multiple layers of semantic information. Both situations are very bad. So, it is very important to scientifically determine the number of topics. The strength of the theme depends on the ranking number. Divide the same group of technologies, calculate the intensity of the same group of technologies in each time window, and analyze the change of theme intensity of the same group of technologies on the time axis.

CNN is a back-propagation network, which performs well in many fields such as image processing and speech recognition. Compared with other standard neural networks in the same layer, CNN has relatively few parameters and requires less training time. This paper applies CNN model to the task of Chinese patent text classification. One is to construct the classic CNN model of patent text classification, and the other is to be an important part of the combined Chinese patent text classification model proposed in this paper.

This paper assumes that the input of attention mechanism is *M* = {*m*_1_, *m*_2_, ⋯, *m*_*n*_}, and the attention value can be calculated by the following formula.

(6) $$\begin{array}{c} \text{score}\left(m_{i}\right)=v^{T}\tanh\left({wm}_{i}+b_{i}\right), \end{array}$$

where *w* is the weight, *b*_*i*_ is the bias term, and score(*m*_*i*_) is the score of the input information; then, use Softmax function to normalize.

Theme intensity indicates the activity of the theme in the current time window. In the same time window, the higher the number of patent texts of this subject, the higher the intensity of the subject, the higher the popularity of this type of patent technology, and the higher the application amount. This document adopts the topic intensity measurement method, and the specific topic intensity calculation formula is as follows:

(7) $$\begin{array}{c} Q\left(Z_{t,k}\right)=\frac{\sum_{d=1}^{M}\theta_{d,k}}{M}. \end{array}$$

*θ*_*d*,*k*_ represents the probability of the *k*th topic in the *d* document, and *Q*(*Z*_*t*,*k*_) represents the intensity of the topic *k* in the current time slice *t*.

A KNN classification method that has been optimised is created by combining the clustering concept. The training set's text is preprocessed before the similarity calculation takes place. To do this, first, extract words and features from the training set of texts, then figure out how much each feature element is worth. Second, until all of the texts in the training set have been calculated, define a text and use it and each text in the training set to determine the similarity. The formula for calculating weight is:

(8) $$\begin{array}{c} w_{kj}=\frac{{tf}_{kj}*\log\left(\left(N/N_{j}\right)+0.01\right)}{\sqrt{\sum_{j=1}^{n}{\left(f_{kj}\right)}^{2}*\log^{2}\left(\left(N/N_{j}\right)+0.01\right)}}. \end{array}$$

*tf*_*kj*_ represents word frequency, and *N* represents the number of all texts in the training text set; *N*_*j*_ indicates the number of texts containing feature item *t*_*j*_ in the training text set.

*T* is used as the input data of convolution layer, that is, the new patent text vector, and convolution operation is carried out on the input new patent text vector *T* by using convolution kernel *w* with size *m* × *k*, and the expression is as follows:

(9) $$\begin{array}{c} c_{i}\in f\left({wT}_{i,i+m+1}+b_{i}\right). \end{array}$$

*T*_*i*,*i*=*m*=1_ represents the extraction of local features from the *i*th line to the *i* + *m* + 1 line of *T*, *f* is a nonlinear transfer function, and *b* represents the offset term.

## 4. Experiment and Results

In the 10 patent folders, 30 invention patent items, 30 utility model patent items, and 40 design patent items are randomly selected, and a total of 1,000 patent items constitute the test set; this training set and test set are used to test the running efficiency and performance of the two classifiers. We evaluate the classification effect of the whole text system by calculating the operation rate, accuracy rate, error rate, and recall rate.

When *K* = 20, the classification data of the optimized KNN algorithm and the traditional KNN algorithm in terms of operation rate, accuracy rate, and error rate recall rate are shown in Figures 3 and 4.

Combining the clustering idea results in an optimised KNN classification algorithm. Before determining similarity, the text from the training set is preprocessed. To accomplish this, first, take words and features out of the training set of texts, and then, calculate the value of each feature element. Second, define a text and use it together with each text in the training set to calculate the similarity until all of the texts in the training set have been calculated. The weight calculation formula is as follows.

How to partition the data is the key topic of task decomposition. After partitioning the data, the size of each section also affects the performance of the classifier. We observe the impact of model classification on large-scale patent classification by changing the modulus and using two splitting methods: random split and prior knowledge split. A comparative study of random partition and prior knowledge partition methods. The results are shown in Tables 1 and 2.

Through the experimental results, we can analyze the different characteristics of random splitting and prior knowledge splitting: the advantage of random splitting is that it keeps the general distribution of the original sample space. With the increase of training set, the module size should be increased correspondingly to achieve the best classification performance. The prior knowledge is well divided according to the clustering distribution of data in the feature space, and each module contains the nearest sample in the space. When the module size is relatively small, these two types of subproblems become completely linear. The excellent performance of subclassifier improves the overall performance of classifier.

The loss function used in this work is the cross entropy function, which is based on entropy and calculates the difference between two probability distributions. It is often used in the classification of neural network types. Avoid excessive sigmoid gradient when calculating loss function. If the problem is too small, input the output of Softmax function to predict the result and calculate the loss value. After the experiment, the dotted lines of the accuracy and loss rates of four Chinese patent text classification models are obtained, as shown in Figures 5 and 6.

As seen in the aforementioned Figure 5, when the test data from the four training models are compared, it is clear that while CNN and LSTM models converge more quickly than this model does, as training times and iterations increase, this model's ability to extract features from patent texts has improved, and its classification accuracy has steadily increased. Compared to CNN and LSTM models, this model's final convergence accuracy is higher. It is clear that LSTM is better suited for serial data, and its accuracy rate of 95% demonstrates that a combined model performs better than a single model.

After the attention mechanism is introduced, a certain amount of computation is needed, and once the input stream increases, the computation will increase exponentially. In addition, compared with the original model, the structure of the model is more complex, resulting in higher initial loss, but the final convergence rate tends to be faster, the recovery rate gradually decreases, and tends to be stable and convergent. According to the probability distribution of document-topic and topic-word extracted by the model in this paper, the topic intensity in each time period is calculated, and the evolution trend of topic intensity in this time period is analyzed. The following is an analysis of various hot topics in rare earth industry, and the specific evolution is shown in Figure 7.

It can be clearly seen from Figure 7 that the theme intensity of each theme changes with the passage of time. From the analysis of the evolution of the intensity of each topic in Figure 7, it can be concluded that the intensity of theme 4 is always high, and the intensity of theme 1 shows a downward trend as a whole, which indicates that the research on magnetic materials has reached a certain technical bottleneck, and the research interest is gradually declining. The content of the subject luminous field shows a big upward trend with the time of subject intensity. In recent years, this technology is a relatively new research field in China. The theme is about the field of glass materials, and the intensity of the theme fluctuates little, which shows that the research in this field is stable.

Aiming at the problems of uneven index quality and high maintenance cost in multi-index retrieval, this paper puts forward the concept of application-oriented dynamic index set, puts forward the index evaluation and optimization mechanism, and constantly optimizes the index structure. This paper describes the principles of conflict and conflict and conflict and invention and uses engineering semantic web tools to solve knowledge and deeply analyze the internal structure of innovative design schemes.

Introducing punitive damages into IP law can break the restriction of criminal sanctions for IP infringement. The introduction of punitive damages in China's IP law can break the restriction of criminal sanctions, but if offenders are to be imprisoned to limit their illegal behavior, it will cause some social problems and public opinion. Regarding the introduction and implementation of punitive damages, China must also distinguish between copyright infringement and patent infringement. Patent infringement mostly occurs in enterprises, which is an important foundation for the development of enterprises. Copyright infringement mostly happens to individuals, and the state should also protect the legitimate rights and interests of individuals according to law and compensate the victims.

## 5. Conclusions

Intellectual property has grown to be an incredibly significant intangible asset and property right for all nations in the age of the information economy. The capacity to create IP frequently determines a company's entire competitiveness and, sometimes, even the economy of a whole nation. This essay examines the restrictions placed on the noncontractual damage principle in the defence of victims' rights and interests based on the judicial application of the punitive damage system and noncontractual damages. A patent text classification experiment was conducted on text data in the computer field, and a Chinese patent text classification system was designed to directly store the obtained Chinese patent text data in the database. This experiment was inspired by deep learning to deal with Chinese text classification and combined with the familiar knowledge of computer field. Additionally, the database's Chinese patent documents have stop words removed and are split. This model's feature extraction function enhances the feature extraction function of patent texts, and classification accuracy is continuously increased. This model finally gets a 95% convergence rate. The optimised KNN classification algorithm, according to experiments, outperforms the conventional KNN classification algorithm.

## Figures and Tables

**Figure 1:** Legal support system.

**Figure 2:** Functional architecture diagram of Chinese patent text classification system.

**Figure 3:** Optimize the preclassification result.

**Figure 4:** Optimized postclassification results.

**Figure 5:** Accuracy line chart of four models.

**Figure 6:** Line chart of loss rate of four models.

**Figure 7:** Evolution trend of hot topic intensity.

**Table 1:** Randomly divide the number of modules and classification accuracy.

Module size	Macro *F*1 (%)
7000	80.687
6000	80.441
5000	80.782
4000	80.649
3000	80.351
2000	80.839
1000	80.339

**Table 2:** Number of prior knowledge partition modules and classification accuracy.

Module size	Macro *F*1 (%)
1000	90.348
800	90.439
600	90.126
400	90.126
200	90.199

## Data Availability

The data used to support the findings of this study are available from the corresponding author upon request.
